# Research on Building Space Model Method Based on Big Data Map Visual Design

**DOI:** 10.1155/2022/3384948

**Published:** 2022-05-11

**Authors:** Qiang Xu, Long He

**Affiliations:** ^1^School of Architecture, Tianjin University, Tianjin 300072, China; ^2^School of Architecture, Inner Mongolia University of Technology, Hohhot, Inner Mongolia 010050, China

## Abstract

In order to explore the architectural space model of design, a visualization method based on big data map is proposed. Referring to the tile pyramid model, a multidimensional aggregation pyramid model (MAP) is proposed, which extends the 2D spatial hierarchical aggregation of tile pyramid to the multidimensional of time/space/attribute and supports the multidimensional hierarchical aggregation of time, space, and attribute. Then, taking spark cluster as the parallel preprocessing tool and HBase distributed database as the persistent storage of map model data, an open-source distributed visualization framework (MAP-Vis) is realized. Then, the BIM model is reconstructed, and a component instance hierarchical splitting strategy based on IFC structure tree is proposed to separate the digital and analog of the original IFC file. The reconstructed IFC model file is transformed into glTF format file, and the dual relationship mapping of geometric space and semantic attributes is completed in the transformation process. Finally, the visibility detection algorithm of BS-AB scene components based on the hierarchical bounding volume (BVH) structure is proposed to eliminate the visibility of building components. The experimental results show that BIMviews is slow to load the IFC file of the experimental object and obtain the model data, with an average of about 40 s, and the Caton is obvious. However, it only takes about 7 s to load glTF file into big data map visualization design by Three.js. It is verified again that glTF format is more suitable for BIM model data than IFC format. The visualization design, display, and interaction based on big data map are based on glTF format. It proves the effectiveness of big data map visualization.

## 1. Introduction

With the maturity and diversification of data acquisition means such as personal intelligent devices, floating car GPS, Internet of things, and social media, the data sources are becoming richer and richer, and the amount of data collected is increasing explosively. These big data with huge volume, stream generation, numerous types, and value contain both space-time and high-dimensional characteristics [1]. Spatiotemporal features refer to data with spatial location and time tag or attribute fields that can reflect spatiotemporal location. High-dimensional feature refers to that the data contain other feature attributes except time and space, and the information law reflected by these attributes is often more valuable for research. Visualization is an important step and means of analyzing and mining spatiotemporal big data, which can directly reflect the patterns and laws contained in the data. The building information model (BIM) provides advanced digital tools and information-sharing platform for the information management of the whole life cycle of construction projects. It solves the problems of information transmission fault and data-sharing difficulties faced by traditional facility engineering and has been widely used in architecture, engineering, construction, and facility management (AEC/FM) [2] (Figure 1). The greatest value of BIM lies in the efficient collaboration between multiple participants and multiple disciplines. With the continuous increase of building scale and the increasing complexity of building information data, its model visualization and massive data management become more and more difficult so that it cannot meet the current BIM localization application requirements of engineering construction information data management, sharing, and synchronization. Obviously, while meeting the needs of multiple users to access anytime and anywhere under different devices and different operating systems, it is particularly important to effectively ensure the integrity semantics of BIM model and data interoperability [3].

## 2. Literature Review

Zhu W. puts forward the general laws and characteristics of the thinking process of architectural creation and combined and summarized the visual expression and design tools [4]. Zhao L. divided the visual media of design into three aspects, drawing, solid model, and digital design, and analyzed how it affected the design information, so as to better complete and express the design [5]. MW Kowalczyk attempts to visualize the architectural design process from the perspective of computer programming [6]. Djari C. systematically summarized the development of relevant factors, information sources, design carriers, and expression tools of visualization technology and theory and discussed the specific application in different stages of the design process, to provide effective visual expression ways for designers in the process of architectural design [7]. Ladlf Su á rez proposed sequence snapshot and model in “time in GIS.” The sequence snapshot model is the simplest spatiotemporal data model at present. It is widely used in various temporal GIS systems. This data model completely stores the state data at different times in the study area so that the objects that have not changed are repeatedly saved, resulting in data redundancy and reducing the use efficiency of the system [8]. Haiyan et al. proposed a ground state correction model on this basis, which only saves the initial state data and the change amount of the change part relative to the initial state in the study area, greatly reducing the data redundancy. However, these models are only simple time simulation and do not really solve the problem of space-time combination [9]. Guan proposed a spatiotemporal composite model for the vector model, which divides space into a set of spatiotemporal composite units representing the same time process [10]. The spatiotemporal object model proposed by Zou Y. introduces the time dimension to make it orthogonal to the two-dimensional space and abstracts the real world into a discrete object set composed of spatiotemporal atoms. This kind of model mainly tends to the spatial change of geospatial entities with time, which is a simple simulation of the spatiotemporal change process of the research object [11]. Fu et al. proposed a three-domain model of space-time. They believed that simply introducing time as a new dimension into the space-time data model could not fully express and display the world, so they organized the space-time data from the perspectives of location, time, and object. With the emergence of object-oriented technology in computer, the real world is abstracted into a set composed of different types of objects (entities), and an object-oriented spatio-temporal data model is established. This model has great advantages in describing complex phenomena [12]. Mehta extended the spatiotemporal atomic structure by using Brisson lattice complex and proposed an object-oriented spatiotemporal data model based on lattice tuples [13].

Based on the current research, a method of map visualization based on big data is proposed. Referring to the tile pyramid model, a multidimensional aggregation pyramid model (map) is proposed, which extends the 2D spatial hierarchical aggregation of tile pyramid to the multidimensional of time/space/attribute and supports the multidimensional hierarchical aggregation of time, space, and attribute. Then, the BIM model is reconstructed, and a component instance hierarchical splitting strategy based on the IFC structure tree is proposed to separate the digital and analog of the original IFC file. The reconstructed IFC model file is transformed into glTF format file, and the dual relationship mapping of geometric space and semantic attributes is completed in the transformation process. Finally, the visibility detection algorithm of BS-AB scene components based on the hierarchical bounding volume (BVH) structure is proposed to eliminate the visibility of building components.

## 3. Visualization Design of Big Data Map

### 3.1. 2D Pyramid Model

In the geographic information system (GIS), the tile map pyramid model is often used for 2D map display. It is a multiresolution hierarchical model. From the bottom to the top, the resolution of pyramid is getting lower and lower. The pyramid contains multiple layers. Each layer is spliced by multiple square tiles, and each tile is composed of pixels (the default resolution is generally 256 × 256 pixels). In order to describe the construction process of the 2D pyramid model more accurately, the following concepts are defined in this study:

(1) Pixels: the pixel is the smallest data unit of the pyramid model; that is, a single pixel in the tile in the tile pyramid level is expressed as
  (1) $$\begin{array}{c} \text{pixel}=\left\{l,x,y,p\right\}, \end{array}$$
where *l* is the hierarchy of the pyramid, *X* and *y* are the spatial range contained in the pixel, and *p* represents the characteristic sampling values within the spatial range corresponding to the pixel, such as aggregate statistical values, such as mean and sum.
(2) Tiles: tiles in the tile pyramid model are a combination of pixels adjacent to space, and the default resolution is 256 × 256 pixels, which is expressed as
  (2) $$\begin{array}{c} \text{tile}=\left\{l,X,Y,\overset{w\times w}{\underset{i=1}{\cup }}\text{pixel}\right\}, \end{array}$$
where *l* is the hierarchy of the pyramid, *X* and *y* are the row and column numbers of the tiles, w is the resolution of the tiles, and the last union represents the set of pixels within the space of the tiles [14].
(3) Pyramid: pyramid is a spatial multiscale model composed of tiles at all levels and is expressed as
  (3) $$\begin{array}{c} \text{pyramid}=\sum_{i=1}^{n}\sum_{j=1}^{M}\sum_{k=1}^{N}\text{tile}\left\{l_{i},X_{j},Y_{k},\overset{w\times w}{\underset{i=1}{\cup }}\text{pixcel}\right\}. \end{array}$$

Based on the above concepts, the construction of the pyramid model also needs corresponding operations to jointly complete the hierarchical aggregation of spatial dimensions. The four basic operations defined are as follows:

(1) Extract operation: it is responsible for mapping each original record to the pixel unit. A pixel may correspond to one or more original records. The extract operation is
  (4) $$\begin{array}{c} \text{Extract}\left(l_{n},\left\{Lon,Lat\right\},w\right)=\text{pixcel}\left\{l_{n},x,y,p\right\},\\ \left\{\begin{array}{c} x=\frac{Lon+180}{360}•2^{l_{n}+r},\\ y=\left(1-\frac{\left(\tan\left(Lat•\pi /180\right)+1/\cos\left(Lat•\pi /180\right)\right)}{\pi }\right)•2^{l_{n}+r-1},\\ r=\log_{2}\;w. \end{array}\right) \end{array}$$
(2) Group operation: it is mainly to establish the corresponding mapping relationship between pixels and tiles, that is, to obtain the specific tiles to which the pixels should belong. The operation formula is
  (5) $$\begin{array}{c} \text{Group}\left(\text{pixcel}\left\{l_{n},x,y,p\right\}\right)=\text{tile}\left\{l_{n},X,Y,\overset{w\times w}{\underset{i=1}{\cup }}\text{pixcel}\right\},\\ \left\{\begin{array}{c} X=\left(\frac{x}{w}\right),\\ Y=\left(\frac{y}{w}\right). \end{array}\right) \end{array}$$
(3) Key value operation: the largest level of tiles and their aggregate data are obtained through group operation. The key can be the quadtree/space filling curve code of the tile, the value is the set of pixels of the tile, and its key value will be converted. The tiles will be stored in the form of key value pairs to establish the foundation for subsequent distributed storage.
(4) Aggregate operation: unlike the group operation, which combines pixels within a single tile, aggregate is the aggregation of tiles between levels. Extract, group, and key value operations obtain the tile set of the largest level of the pyramid. Next, they need to aggregate up level by level to get the tiles of each level and finally get the pyramid model. The aggregate operation formula is
  (6) $$\begin{array}{c} Agg\left(\text{tile}\left\{l_{n},X_{2i},Y_{2i},\overset{w\times w}{\underset{i=1}{\cup }}\right\}\text{pixel}\right),\\ \left(\text{tile}\left\{l_{n},X_{2i},Y_{2i+1},\overset{w\times w}{\underset{i=1}{\cup }}\right\}\text{pixel}\right),\\ \left(\text{tile}\left\{l_{n},X_{2i+1},Y_{2i},\overset{w\times w}{\underset{i=1}{\cup }}\right\}\text{pixel}\right),\\ \left(\text{tile}\left\{l_{n},X_{2i+1},Y_{2i+1},\overset{w\times w}{\underset{i=1}{\cup }}\right\}\text{pixel}\right)=\left(\text{tile}\left\{l_{n-1},X_{i},Y_{i},\overset{w\times w}{\underset{i=1}{\cup }}\right\}\text{pixel}\right). \end{array}$$

### 3.2. Multidimensional Aggregation Pyramid Model

The multidimensional aggregation pyramid (map) model is a spatiotemporal multidimensional hierarchical aggregation model based on the traditional tile pyramid model. Among them, the temporal dimension and spatial dimension belong to positioning features. The whole composed of the two identifies a spatiotemporal unit and serves as the key of the spatiotemporal unit. The discrete attribute dimension aggregation tree is value, and the two correspond in the form of key value pair. In this way, while realizing spatiotemporal aggregation, attribute dimensions are also aggregated, and a multidimensional spatiotemporal aggregation pyramid model containing space, time, and attribute dimensions is obtained [15].

(1) Aggregation tree (faa_tree): attribute aggregation tree is a tree structure formed by aggregating each dimension unit of the attributes of spatiotemporal objects, which simplifies the actual storage space with the result of breadth first traversal. Obtain a fixed length 1-dimensional array that can be stored structurally, and the formula is
  (7) $$\begin{array}{c} faa\_\text{tree}=\left\{a_{\text{all}},a_{1},a_{2},\ldots ,a_{n}\right\}, \end{array}$$
where *a*_all_, *a*_1_, *a*_2_,…, *a*_*n*_. The node array sequence is obtained by traversing the attribute aggregation tree according to the hierarchy. Compared with tree structure, the fixed length array structure provides great convenience for subsequent storage and processing.
(2) Spatiotemporal pixel (st pixel): different from the zero-dimensional characteristics of pixels in 2D map tiles, spatiotemporal pixels are a one-dimensional structure, a container for attribute dimensional information, and the smallest data unit of the map model. Spatiotemporal pixels extend the connotation of the concept of tile pyramid pixels. In addition to the range of spatial coordinates, they also add time scale coordinates. The formula is
  (8) $$\begin{array}{c} ST-\text{pixel}=\left\{l,x,y,t,faa\_\text{tree}\right\}, \end{array}$$
where *t* represents the scale coordinates of the preset time granularity and tree is the attribute aggregation *faa*_tree, which is the real source of visual content.
(3) St tile: the concept of spatiotemporal tile is like that of the 2D model, which is composed of spatiotemporal pixels. Spatiotemporal tiles contain spatiotemporal pixels. Spatiotemporal pixels mount the attribute dimension aggregation tree to form a spatiotemporal cube that can realize hierarchical aggregation. Spatiotemporal tile is the basic unit of map model display. It is a 5-tuple, defined as
  (9) $$\begin{array}{c} ST-\text{tile}=\left\{L,X,Y,T,\text{Tile}\_faa\right\}, \end{array}$$
where *l* is the level of pyramid, *X* and *y* are the row and column numbers of tiles, and *T* represents the scale coordinates with preset time granularity, and Tile _faa formula is
  (10) $$\begin{array}{c} \text{Tile}\_faa=\left\{A_{\text{all}},A_{1},A_{2},\ldots ,A_{n}\right\}, \end{array}$$
where *A*_all_, *A*_1_, *A*_2_,…, *A*_*n*_ is the attribute aggregation tree at tile level obtained by accumulating the subscripts corresponding to the array sequence faa_tree of attribute aggregation trees of each pixel in the tile.

It can be seen from (10) that the defined space-time tile is no longer a two-dimensional plane in concept, so the basic operations in the two-dimensional need to be further expanded.

(1) Extract operation: in addition to extracting geographic location information, it is also necessary to extract time information and attribute dimensions, generate attribute aggregation tree, and list them in order. The operation is
  (11) $$\begin{array}{c} \text{Extract}\left(l,Lon,Lat,w\right)=ST-\text{pixel}\left\{l,x,y,t,faa\_\text{tree}\right\}. \end{array}$$
(2) Group operation: there are two steps. The first step is mainly to establish the corresponding mapping relationship between spatiotemporal pixels and spatiotemporal tiles, that is, to obtain the specific tiles to which the pixels should belong, so as to locate not only in space but also in time. The formula is
  (12) $$\begin{array}{c} \text{Group}\left(ST-\text{pixel}\left\{l,x,y,t,faa\_\text{tree}\right\}\right)=ST-\text{tile}\left(\left[l_{n},X,Y,T,\text{Tile}\_faa\right]\right), \end{array}$$
where *t* and T represent the time limit required for group operation. Therefore, the spatiotemporal unit to which each pixel belongs can be found through (12), and the spatiotemporal pixels can be mapped to specific spatiotemporal tiles.
The second step of group operation is to reduce all spatiotemporal pixels mapped to the same spatiotemporal tile and aggregate all pixels in the tile under the same time granularity and the same geographical range. At the same time, the aggregation tree tile of the spatiotemporal Tile_faa st tile is the accumulation of the corresponding positions of the 1-dimensional fixed length array faa_tree of all spatiotemporal pixels, and the formula is
  (13) $$\begin{array}{c} ST-\text{Tile}\_faa=\sum_{i=1}^{N=n}ST-\text{pixel}.faa\_\text{tree}. \end{array}$$
(3) Key value operation: split tile_. For each node in FAA, the node is jointly encoded with the quadtree and time *t* of the tile to generate the key. Then, take the pixel set corresponding to each node as a value to generate a key value pair. The true meaning of the key value operation is the statistical result of the event of an attribute node within the tile space within the time period *T*.
(4) Aggregate operation: it needs to be limited to the same time *t*, that is, aggregate the tiles after key valued and finally obtain the multidimensional pyramid model. The formula is
  (14) $$\begin{array}{c} Agg\left(ST-\text{tile}\left(l_{n},X_{2i},Y_{2i},T,\text{Tile}\_faa\right)\right),\\ ST-\text{tile}\left(l_{n},X_{2i},Y_{2i+1},T,\text{Tile}\_faa\right),\\ ST-\text{tile}\left(l_{n},X_{2i+1},Y_{2i},T,\text{Tile}\_faa\right),\\ ST-\text{tile}\left(l_{n},X_{2i+1},Y_{2i+1},T,\text{Tile}\_faa\right)=ST-\text{tile}\left(l_{n-1},X_{i},Y_{i},T,\text{Tile}\_faa\right). \end{array}$$

### 3.3. Scenario Management Strategy

In the actual rendering process, there are usually tens of thousands of building components in a rendered scene, and the network bandwidth, memory capacity, and rendering performance are often limited. If all components in the rendered scene are rendered indiscriminately, it will cause great performance sales to GPU and reduce the efficiency of graphics rendering. Therefore, it is very important to optimize the organization, management, and scheduling of rendering scenes. There are many solutions for the management and optimization of rendered scenes, such as visibility culling, region of interest setting, LOD index structure, and batch call rendering [16].

The view range of browser model data is composed of viewpoint position and view cone, which is usually only a part of the whole rendered scene. Therefore, the organization and management of rendering scene through visibility culling is a widely used scene management method. Visual cone culling, back face culling, and occlusion culling are three widely used visibility culling technologies. The technical comparison is shown in Figure 2.

The back culling is carried out in the rasterization stage. It improves the rendering performance by culling the pieces back to the viewpoint. It is a visibility culling algorithm supported by the native OpenGL. Occlusion elimination can eliminate invisible objects blocked by visible objects. Although it can reduce the performance overhead of rendering pipeline and GPU, it is implemented based on hardware and needs to collect the location information of occluded objects and occluded objects, which occupies CPU resources. Visual cone culling exists in many real-time renderings. It is used to cull polygons or objects outside the visual cone view and render only the geometric graphics within the visual cone view, to improve the efficiency of graphics rendering. Relatively speaking, the visual cone elimination algorithm is suitable for the organization and management of rendered scenes [17]. In this study, BSphere volume and AABB box collision detection algorithm are introduced to construct the visual cone elimination algorithm based on BVH.

### 3.4. Experimental Method and Process

#### 3.4.1. Model transformation

The original IFC file usually contains geometric information (spatial position and spatial relationship, etc.) and nongeometric information (attribute type and material map, etc.), and in the process of model conversion, it will often cause the lack of architectural object semantic attribute information, resulting in the lack of model information integrity. Therefore, it is necessary to separate the BIM model from the digital model and store and load the geometric space information and semantic attribute information separately, to ensure the integrity and semantics of the BIM model. IFC organizes and manages the building and component information of the BIM model in the form of the tree structure. Each building component instance is a node on the IFC structure tree, and each node has spatial or attribute relationships such as inclusion and association with its parent node or through its parent node and other child nodes. For example, each IFC wall instance is included in the IFC wall parent node as a child node, and similarly, the IFC wall parent node is included in the IFC building element as a child node, which is associated with the IFC door. By recursively accessing each node of the IFC structure tree and exporting the geometric attribute information of building component instances or other BIM scene information hierarchically, it can not only effectively manage IFC files and reduce IFC data redundancy but also lay a foundation for component batch rendering.

BIM server provides IFC file management, data analysis, formatted output, and other functions. This study will also traverse and retrieve the hierarchical relationship of the whole building model through the BIM server and split the building model into corresponding IFC model files and JSON text files through recursive access to the IFC structure tree. IFC model files store BIM spatial and geometric information, while JSON text files store BIM attribute and type information [18]. The digital analog separation process is shown in Figure 3.

In the past research studies, there are many solutions to convert IFC format files into GLTF format files. Select OBJ files as the intermediate format. First, call the IFC convert tool in the Ifc open shell library to convert IFC files into OBJ files and then convert OBJ into GLTF format files through the obj2gltf tool launched by AGI (analytical graphics, Inc.), so as to realize the overall conversion from IFC to glTF. By calling Revit API and inheriting IExternal Command and IExternal Application interfaces, this study constructs IFC glTF conversion framework based on c# language and realizes glTF model file output through Revit2gltf. The data conversion process is shown in Figure 4 [19].

Usually, in the process of BIM model transformation, it is necessary to complete the spatial relationship mapping from geometric information to WebGL. This is because the component position coordinate information in IFC file is defined by IfcLocalPlacement attribute, which usually adopts the local coordinate system, while WebGL is the global coordinate system. Therefore, to establish the connection between IFC model components and WebGL camera, coordinate system space transformation must be carried out, mainly including model transformation and visual transformation. The coordinate transformation from the local coordinate system to the world coordinate system is the transformation of spatial geometry by translation, scaling and rotation alone or in combination [20]. Considering that the Cartesian coordinate system adopts the right-hand rule, take the *z*-axis as an example, as shown in Figure 5.

Usually, a point *V*(*x*, *y*, *z*, 1) in space will pass through 4×4 matrix *M* transformation in (15) to get a new point *V*′(*x*′, *y*′, *z*′, 1):

(15) $$\begin{array}{c} \left[\begin{array}{cccc} a & b & c & d\\ e & f & g & h\\ i & j & k & l\\ m & n & o & p \end{array}\right]\times \left[\begin{array}{c} x\\ y\\ z\\ 1 \end{array}\right]=\left[\begin{array}{c} x^{\prime }\\ y^{\prime }\\ z^{\prime }\\ 1 \end{array}\right]. \end{array}$$

If a vertex *V*_Local_(*x*, *y*, *z*, 1) in the local coordinate system translates the distance *T*_*x*_, *T*_*y*_, *T*_*z*_ on the *x*-axis, *y*-axis, and *z*-axis, respectively, to obtain *V*_Global_(*x*′, *y*′, *z*′, 1)=*V*_Local_(*x*+*T*_*x*_, *y*+*T*_*y*_, *z*+*T*_*z*_, 1), and substituting it into (15), we can obtain the translation matrix, i.e.,

(16) $$\begin{array}{c} T=\left[\begin{array}{cccc} 1 & 0 & 0 & T_{x}\\ 0 & 1 & 0 & T_{y}\\ 0 & 0 & 1 & T_{z}\\ 0 & 0 & 0 & 1 \end{array}\right]. \end{array}$$

If the point is scaled with the origin as the base point and *S*_*x*_, *S*_*y*_, and *S*_*z*_ times are scaled in the *x*-axis, *y*-axis, and *z*-axis directions, respectively, the point *V*_Global_(*x*′, *y*′, *z*′, 1)=*V*_Local_(*x*+*S*_*x*_, *y*+*S*_*y*_, *z*+*S*_*z*_, 1) will be obtained, which can be substituted into (15) to obtain the scaling matrix, i.e.,

(17) $$\begin{array}{c} S=\left[\begin{array}{cccc} S_{x} & 0 & 0 & 0\\ 0 & S_{y} & 0 & 0\\ 0 & 0 & S_{z} & 0\\ 0 & 0 & 0 & 1 \end{array}\right]. \end{array}$$

If the figure rotates around the *Z*-axis, as shown in Figure 6, the *Z* value transformation can be ignored because the *Z* value remains unchanged. At this time, set *R* as the distance from the origin *o* to the point *V*_Local_(*x*, *y*, *z*). *α* is the angle the *X*-axis rotates to this point. According to the trigonometric function equation, the rotation matrix when the point *V*_Local_(*x*, *y*, *z*) rotates at angle *ß* around the *Z*-axis can be obtained, i.e.,

(18) $$\begin{array}{c} R_{z}=\left[\begin{array}{cccc} \cos\;\beta_{z} & -\sin\;\beta_{z} & 0 & 0\\ \sin\;\beta_{z} & \cos\;\beta_{z} & 0 & 0\\ 0 & 0 & 1 & 0\\ 0 & 0 & 0 & 1 \end{array}\right]. \end{array}$$

Similarly, the rotation matrix *R*_*x*_ when rotating angle B around the *X*-axis and the rotation matrix *R*_*y*_ when rotating angle *ß* around the *Y*-axis can be obtained.

To sum up, the geometric information of IFC model file can be transformed into the spatial coordinate system through (19) to complete the spatial relationship mapping from component geometric information to WebGL, that is,

(19) $$\begin{array}{c} V_{\text{Global}}=V_{\text{Local}}\times \left(T\times s\times r\right), \end{array}$$

where *R*=*R*_*x*_*R*_*y*_*R*_*z*_ is the rotation conversion matrix when the vertex rotates around the coordinate axis. After digital analog separation and data conversion, glTFmodel file and JSON semantic attribute file are introduced into the same scene object through the constructor “Loader” in Three.js to complete the loading of geometric model and semantic attribute information in WebGL [21].

#### 3.4.2. Scene Management

Visual cone culling uses the spatial correlation in the rendered scene to judge whether the scene model is inside or intersecting with the visual cone. The viewing cone itself is usually composed of 6 cutting planes, and the right section of the cutting plane is shown in Figure 6. The opening angle is in the vertical direction of the apparent cone. *Dn* and *Df* are the distances from the viewpoint to the near clipping plane and the far clipping plane, respectively. *Hn* and *Hf* are the heights of the near clipping plane and the far clipping plane, respectively.

Suppose the aspect ratio of the camera is *k* and a vertex P (XO, Jo, Zo) is on the side of the right clipping plane. According to the geometric relationship, the distance between the vertex and the right clipping surface can be calculated through equation (6), to judge the spatial relationship between the vertex and the right clipping surface, i.e.,

(20) $$\begin{array}{c} d=\frac{\left|x_{0}+k\;\tan\theta /2z_{0}\right|}{\sqrt{1+k^{2}\tan^{2}\left(\theta /2\right)}}. \end{array}$$

If *d* < 0, the apex is outside the visual cone. If *d* ≥ 0, the apex is inside the visual cone. This is because when the clipping space changes, the left- and right-hand coordinate system changes, and the normal vector of the clipping surface points to the viewing cone. According to the spatial relationship between all vertices of a component and the clipping surface, it can be determined whether the whole component and the viewing cone have an inclusion, intersection, or separation relationship, to determine whether to load and render the component.

*(1)* BVH-based visibility detection algorithm for BS-AB scene components: using the spatial data structure with hierarchical structure to organize the scene and build a bounding box approximate description component with slightly large volume but relatively simple geometric features is a favorable way to solve the low efficiency of linear array traversal in complex scenes and the difficulty of visual cone intersection test of complex components. Hierarchical bounding volume (BVH) is a commonly used spatial data structure. It organizes and manages the objects in the scene in a hierarchical tree structure based on spatial information, including internal nodes and leaf nodes from the root node down.

Therefore, the BVH structure tree can be created according to the IFC component tree. Here, the cone scene is regarded as a root node, and each Ifc Building Element (such as IfcWall and IfcDoor) is placed in the internal node as a category; then, the family under each category is the leaf node. When there are still different components in the leaf node, continue to build the BVH tree according to the family and family type until the leaf node contains family instances. The purpose of adding enclosures in the scene is to filter the geometry outside the enclosure through accurate collision detection. Commonly used bounding bodies include BSphere body and AABB box. Bsphere volume algorithm is based on the sphere radius *R* and the distance *d* from the sphere center to the cutting surface of the viewing cone. If *d* < *r*, the sphere is separated from the visual cone without loading. If |d|<*r*, the sphere intersects with the visual cone for loading. If *d* > *r*, the sphere is loaded in the viewing cone, and its structure is shown in Figure 7. The AABB box algorithm is based on the distance between the vertex of the bounding box and the cutting surface of the viewing cone. Whether to load the bounding box is determined by judging whether the vertex of the bounding box is in the viewing cone or whether the connecting line between two points passes through the viewing cone. Its structure is shown in Figure 8.

When collision detection is performed between the visual cone and the hierarchical bounding body, BSphere predetection is performed first, and recursive access is performed to each node from the root node in turn. The separated internal nodes and leaf nodes are eliminated, and the leaf nodes contained in the internal nodes and the internal nodes intersecting with the visual cone are loaded. In addition, the leaf nodes that still intersect the visual cone in the internal nodes intersecting the visual cone are detected by AABB box, and the bounding boxes that are separated from the visual cone are eliminated. Based on ensuring the efficiency of visual cone elimination, this algorithm not only reduces the performance overhead of rendering pipeline but also improves the accuracy of visual component detection [22].

Sphere structure and intersection test are simple, but the tightness is too poor. Although AABB box supports dynamic update and detection is more accurate, the update efficiency is too low. Therefore, this study proposes to carry out sphere predetection on scene components, eliminate rough and loose components, and then further screen through AABB box detection to quickly achieve the optimal detection results.

## 4. Experiment and Result Analysis

In order to verify the effectiveness of model transformation strategy and scene management strategy, this study collects 10 experimental data of building scene composition from the open IFC model repository and BIM model databases for example verification. This example verifies that it is configured as Intel(R) Core (TM) i7-8700@3.20GHZ six core processor, 16 GB memory, NVIDIA GeForce GTX 1060 graphics card, and notebook computer with 64 bit Windows10 operating system is implemented based on Chrome browser and Three.js framework. The IFC version of all test data in the experiment is IFC2X3, as shown in Table 1.

### 4.1. Effectiveness Analysis of Model Transformation Strategy

In this study, glTF is proposed as the target format of model transformation to realize network loading. In this study, the model transformation experiment of IFC model file without semantic attribute is carried out. It can be seen from Figure 8 that, as the volume of model files increases, the volume of glTF increases slowly, while the growth of obj is larger and much larger than that of glTF files. This is because after digital to analog separation and format conversion of the original IFC file, only a small amount of information is stored in the glTF file, while most of the information is stored in the bin file.

It can be seen from Figure 9 that although the overall file size and conversion time of the converted model are different due to different architectural scenes, the compression rate of gLTF format is more than 90%, which has obvious compression advantages compared with obj format. Therefore, taking gLTF as the target, the format of model conversion is effective to reduce the loading of 3D model data, and it will also be more conducive to the rapid loading of 3D model data on the web.

### 4.2. Effectiveness Analysis of Scenario Management Strategy

Aiming at the problem of low rendering frame rate caused by poor visibility detection effect of scene components, this study proposes to use BS-AB scene component visibility detection algorithm based on BVH to detect and eliminate the visibility of building components. In this study, Medel 10 is taken as the experimental object, and 10 cone scenes with the same angle and the same viewpoint but different distances between the viewpoint and the model are set, as shown in Figure 10. Then, in different cone scenes, the performance is compared with other rendering systems in terms of FPS value and single rendering time, to verify whether this strategy is effective for scene visual component management.

In the experiment, the version of BIMviews that BIMServer depends on is BIMServer1.5.88. Chrome web browser is a 64 bit version of 84.0.4147.89. During the experiment, start the FPS mater in the rendering listener of Chrome browser to monitor the rendering area of 3D scene. Use the stats.js library to monitor the rendering time of the scene area. In addition, BIMviews load IFC model files, and other methods load glTF files.

The experimental results are shown in Figures 9–14. It can be seen from Figures 11 and 12 that, as the distance between the viewpoint and the model decreases, the number of components in the visual cone decreases, and the overall FPS value is gradually increasing, but the increase of the other two methods is small and unstable. After Distance 5, the number of components in the visual cone is greatly reduced. The visual cone elimination effect of this method is obvious, and the rendering frame rate increases steadily. It can be seen from Figure 14 that, before Distance 5, there is little difference in the single rendering time of the two methods, but after Distance 5, the rendering time of the method used in this study decreases significantly. Through experimental comparison, the feasibility of the BS-AB scene component visibility detection algorithm and the effectiveness of the scene management strategy are verified, which can meet the smooth needs of BIM model data network visualization. In addition, during the experiment, it was found that BIMviews were slow to load the IFC file of the experimental object and obtain the model data, with an average of about 40 s, and the Caton was obvious. However, it only takes about 7 s to load the glTF file to the complete display of the big data map visualization design by using Three.js. It is verified again that the glTF format is more suitable for the display and interaction of BIM model data based on the big data map visualization design than the IFC format.

## 5. Conclusion

The visibility of scene components is eliminated by BS-AB scene component visibility detection algorithm based on BVH. The experimental results show that this method greatly reduces the amount of BIM model data, improves the detection accuracy of visual components of the model, and has a good effect of web model loading and rendering. The visibility of components (e.g., building models) cannot be detected by different methods, but the visibility of components (e.g., building models) cannot be detected. The follow-up work will start with LOD and occlusion elimination algorithm to further optimize the performance overhead of rendering pipeline and GPU after rendering scene visual cone elimination.

## Figures and Tables

**Figure 1:** Big data map visual design.

**Figure 2:** Comparison of common visibility culling techniques in rendering process.

**Figure 3:** Digital analog separation process.

**Figure 4:** Data conversion process.

**Figure 5:** Schematic diagram of translation, zoom, and rotation of spatial graphics.

**Figure 6:** Section of the right cutting surface of the cone.

**Figure 7:** Schematic diagram of sphere hierarchical bounding box tree structure. (a) Surround scene components with spheres. (b) Hierarchy tree.

**Figure 8:** Size of the converted model file.

**Figure 9:** BIMServer FPS.

**Figure 10:** Model conversion results.

**Figure 11:** BS-AB FPS.

**Figure 12:** Three. js FPS.

**Figure 13:** Three.JS rendering time.

**Figure 14:** BS-AB rendering time.

**Table 1:** Experimental test dataset.

Model ID	Model name	Size (MB)
1	231110AC11-institute-var-2	2.705
2	Autodesk_hospital_parking garage	6.110
3	20191126AZUMA9	10.001
4	Glodon building	27.315
5	HITOS_070308	61.127
6	PUIH-second phase	77.878
7	Humanized office building	90.514
8	Nihewan visitor center	116.766
9	TJ-taoy uanju-complex-architecture	171.011
10	Shr-office-building-structure	303.608

## Data Availability

The labeled dataset used to support the findings of this study are available from the corresponding author upon request.
